The article "The Effect of Gefitinib on Treatment Necessity and Prognosis of NSCLC Patients with Early EGFR Mutations" was published in 2022. Journal: Contrast Media Mol Imaging.

# The Effect of Gefitinib on Treatment Necessity and Prognosis of NSCLC Patients with Early EGFR Mutations

**DOI:** 10.1155/2022/2228744

**Published:** 2022-10-11

**Authors:** Ruiqiang Song, Yanbo Cheng, Tianxi Zheng

**Affiliations:** Department of Thoracic Surgery, The Third People's Hospital of Zhengzhou, Zhengzhou 450000, China

## Abstract

**Objective:**

To investigate the need for and prognostic impact of gefitinib on the treatment of patients with early-stage epidermal growth factor receptor (EGFR) mutated non-small-cell lung cancer (NSCLC).

**Methods:**

Clinical data of patients with stage IB-IIA non-squamous non-small-cell lung cancer admitted to our thoracic surgery department from January 2020 to January 2022 were collected, and a total of 94 cases were included, divided into 44 cases in the control group (EGFR mutation-negative) and 50 cases in the experimental group (EGFR mutation-positive (including those on medication (19 cases) and those not on medication (31 cases)) according to the outcome of EGFR mutation. To evaluate the necessity and prognostic effect of gefitinib in the treatment of NSCLC patients with early EGFR mutations.

**Results:**

The lung cancer recurrence rate in the experimental group (66.00%) was higher than that in the control group (40.91%), and the difference was statistically significant (*χ*^2^ = 5.937, *P*=0.015); in the subgroup analysis of the experimental group samples, the pharmacological intervention of gefitinib had a significant effect on lung cancer recurrence (*χ*^2^ = 7.797, *P*=0.005), and the proportion of lung cancer recurrence in patients not taking the drug (80.65%) was significantly higher than in the drug-taking group (42.11%); the median survival time was 53.6 months using EGFR mutation type as the study factor, with a statistically significant difference in change in 5-year survival rate for EGFR mutation type (*χ*^2^ = 6.095, *P*=0.047) and the lowest 5-year survival rate for subjects with EGFR mutation type Exon 20 T790M.

**Conclusion:**

Patients with early gene drive positive lung adenocarcinoma are significantly more likely to recur and metastasise and have shorter survival times in the absence of pharmacological intervention.

## 1. Introduction

With the deterioration of the living environment caused by industrialisation and the surge of social pressure, lung cancer, i.e. primary bronchial lung cancer, has become the most common malignant tumour in China in terms of incidence and mortality rate [1, 2], and most of the patients are detected during the physical examination as there are often no accompanying symptoms in the early stage or the symptoms are not typical. However, due to the poor awareness of health check-ups among some people, the large economic disparity across the country and the lack of timely detection and diagnosis of patients in less developed areas due to various factors, the vast majority of patients in China are diagnosed at an advanced stage of lung cancer. Patients with advanced lung cancer are often accompanied by metastases to distant organs with large tumour sizes and multiple lymph node metastases [3]. Liver, bone, and brain metastases are common in patients with advanced lung cancer, and when brain metastases occur, the median survival time (overall survival, OS) of patients is only 1 month if they are not treated effectively [4]. When the disease is at an early stage, surgical resection can be used to obtain a longer survival time, but when the disease is at an advanced stage, the patient's general condition is often poorer, immunity is relatively lower, and tolerance to systemic chemotherapy is reduced [5], so treatment of patients with advanced lung cancer is relatively difficult, the disease control rate is significantly lower, and the patient's prognosis is poor [6, 7]. According to the histological type, lung cancer can be divided into non-small-cell lung cancer (NSCLC) and small-cell lung cancer (SCLC). Of these, non-small cell lung cancer is the most common, accounting for approximately 85% of all types [8]. Non-small cell lung cancer includes adenocarcinoma of the lung, squamous cell carcinoma of the lung, and large cell carcinoma, with adenocarcinoma of the lung being the most common of these many classifications. Patients with non-small-cell lung cancer, especially those with lung adenocarcinoma, are prone to mutations in a variety of driver genes, including epidermal growth factor receptor (EGFR), anaplastic lymphoma kinase (ALK), and other mutations. EGFR mutations are the most common type of mutation, accounting for about 50% of all mutations [9, 10], and they have been the most intensively studied. EGFR is a member of the ErbB family of transmembrane proteins, which includes EGFR (ErbB-l), HE R2 (ErbB-2), Her3 (ErbB-3), and Her4 (ErbB-4). Each protein in the ErbB family comprises 3 parts, namely the extracellular region, the hydrophobic transmembrane segment, and the intracellular region. The extracellular region is responsible for binding to extracellular ligands, while the intracellular region is the one containing the tyrosine kinase domain [11]. EGFR can bind to seven ligands, and growth factors bound to EGFR cause a large conformational change in the extracellular region, leading to a dimerisation arm in the second structural domain of the extracellular region. Two ligand EGFR complexes bind to form a back-to-back dimer in which the ligand is located on the opposite side of the aggregate. Upon ligand binding, the EGFR intracellular kinase structural domain forms an asymmetric homodimer, and the dimer activates the carboxy-terminal lobe of the kinase to interact with the amino-terminal lobe of the receptor kinase, leading to its metastable stimulation. Signalling pathways downstream of the protein, including PI3K/AKT/mT0R, RAS/RAF/MAPK, and JAK/STAT, can be activated, thereby regulating cell growth, proliferation, differentiation, and apoptosis [12]. Tumourigenesis can occur when EGFR has altered abnormally, and these alterations include EGFR protein overexpression, increased gene copy number (gene amplification and multimerisation), and mutations.

The article "The Effect of Gefitinib on Treatment Necessity and Prognosis of NSCLC Patients with Early EGFR Mutations" was published in 2022. Journal: Contrast Media Mol Imaging.

Since the successful treatment of lung cancer with the first generation of EGFR inhibitors, a new chapter in targeted therapy for lung cancer has been opened, and targeted therapy has led to improved survival rates for many patients with intermediate to advanced NSCLC [13, 14]. In recent years, there has been a surge in the number of patients with small lung nodules and, consequently, the detection of early-stage lung cancer. Do patients with EGFR mutation-positive early-stage lung cancer require postoperative adjuvant targeted therapy? It has been suggested that patients with EGFR-driven stage IB-IIA high-risk factors and stage IIB-IIIA patients require postoperative chemotherapy and octreotide adjuvant therapy and can benefit significantly [15, 16]. However, what is the therapeutic effect of postoperative adjuvant therapy with EGFR inhibitors in patients with stage IB-IIA lung cancer? Is there a survival difference? As such reports are scarce, the aim of this study was to investigate the impact of pharmacological intervention for EGFR mutations in early-stage lung cancer on recurrence and prognosis in patients with NSCLC in order to find strong scientific evidence to support clinical decision-making.

## 2. Materials and Methods

### 2.1. Clinical Information

The clinical data of patients with stage IB-IIA non-squamous non-small-cell lung cancer admitted to the Department of Thoracic Surgery of our hospital from January 2020 to January 2022 were collected. 94 cases were included, including 41 males and 53 females, 55 cases under 60 years of age, and 39 cases over 60 years of age. The patients were divided into 44 cases in the control group (EGFR mutation-negative) and 50 cases in the experimental group (EGFR mutation-positive (including those on medication (19 cases) and those not on medication (31 cases)) according to the results of EGFR mutation. Tissue sources included mainly surgical specimens, lung puncture biopsies, bronchoscopic biopsies, lymph node puncture biopsies, and metastatic site biopsies. All EGFR genetic tests were performed by direct sequencing. Clinical staging included physical examination, haematology, enhanced ping scan CT or PET-CT of the chest, bronchoscopy, ultrasound of the neck and abdomen, MRI of the brain, and bone scan. The stage I NSCLC was determined using the 7th edition of the American Joint Committee of Cancer (AJCC) TNM staging.

The article "The Effect of Gefitinib on Treatment Necessity and Prognosis of NSCLC Patients with Early EGFR Mutations" was published in 2022. Journal: Contrast Media Mol Imaging.

### 2.2. Selection Criteria

1. Patients with postoperative pathological diagnosis of lung adenocarcinoma and pathological stage IB-IIA, postoperative genetic testing is routinely performed; (2) all patients were first treated in our hospital and had not undergone any other tumour-related treatment before systematic treatment in our hospital; (3) no previous history of malignancy, diabetes mellitus, immune system-related diseases or other serious medical comorbidities.

### 2.3. Method

  2.3.1 Patients' gender, age, ethnicity, past history, smoking history, drinking history, family history, pathological features, and EGFR test results were recorded, and the time and location of tumour recurrence and survival time were recorded in detail during the follow-up.
  2.3.2 Experimental group: patients were recommended to take oral targeted drug therapy (gefitinib) after surgery on a voluntary basis; control group: no targeted drug therapy after surgery, and both groups were strictly followed up.

### 2.4. Statistical Analysis

The data were compiled and analysed using SPSS25.0 statistical software. The data were expressed as “mean ± standard deviation,” and the *t*-test for independent samples was used for comparison between groups, and the *t*-test for paired samples for comparison within groups; the count data were expressed as “*n* (%),” and the chi-square test was used; Kaplan–Meier survival analysis was performed to analyse the survival rate and survival time of the experimental and control groups; the statistical results were judged by *α* = 0.05, and *P* < 0.05, which was statistically significant.

## 3. Results

### 3.1. Clinical Characteristics

The clinical characteristics of the 94 patients enrolled showed a significant difference in the occurrence of lung cancer by gender (*χ*^2^ = 9.148, *P*=0.002), with a significantly higher percentage of lung cancer recurrence in women (67.92%) than in men (36.59%); there was a significant difference between smoking or not for lung cancer recurrence (*χ*^2^ = 7.251, *P*=0.007), with a significantly higher proportion of lung cancer recurrence among smokers (71.05%) than among nonsmokers (42.86%). In contrast, age, history of alcohol consumption, and family history were not significantly different for lung cancer recurrence (*P* > 0.05) (Table 1).

The article "The Effect of Gefitinib on Treatment Necessity and Prognosis of NSCLC Patients with Early EGFR Mutations" was published in 2022. Journal: Contrast Media Mol Imaging.

### 3.2. Recurrence Rate and Site of Recurrence

There was a significant difference in the recurrence rate of lung cancer in the experimental group (66.00%) than in the control group (40.91%) (*χ*^2^ = 5.937, *P*=0.015); in the subgroup analysis of the experimental group samples, there was a significant effect of gefitinib drug intervention on lung cancer recurrence (*χ*^2^ = 7.797, *P*=0.005), and the proportion of lung cancer recurrence was significantly higher in patients not taking the drug (80.65%) than The proportion of lung cancer recurrence in the samples in the drug-taking group (42.11%) was significantly higher (Table 2).

Among the three types with higher mutation frequency, Exon 19 deletion, Exon 20 T790M, and Exon 21 L858, there was a significant difference between different mutation types and metastatic sites (*χ*^2^ = 18.504, *P*=0.005), with a higher percentage of bone metastases (68.18%) occurring in Exon 19 deletion and a higher percentage of brain metastases (56.00%) in Exon 20 T790M had a higher percentage of brain metastases (56.00%) (Table 3).

### 3.3. Effect of Pharmacological Intervention on 5-Year Survival

Using pharmacological interventions as a study factor, the results showed a median survival time of 60.7 months, and the results of the log-rank test showed significant differences between the different experimental subgroups for the change in 5-year survival for follow-up time (months) (*χ*^2^ = 6.791, *P*=0.034 < 0.05) (Tables 4 and 5) (Figure 1).

### 3.4. Impact of EGFR Mutation Type on 5-Year Survival Rate

EGFR mutation type as a study factor showed a median survival time of 53.6 months, and the results of the Log Rank test showed a significant difference in the 5-year survival rate for follow-up time (months) between EGFR mutation types (*χ*^2^ = 6.095, *P*=0.047 < 0.05), with EGFR mutation type Exon 20 T790M subjects had the lowest 5-year survival rate (Tables 6 and 7) (Figure 2).

## 4. Discussion

Lung cancer is the highest mortality rate among malignant tumours in China, with an annual incidence of 53.57/100,000, a standardised rate of 25.34/100,000 for the Chinese population, and a mortality rate of 45.57/100,000 for lung cancer in the same period [17]. Currently, lung cancer accounts for 20.48% of the incidence rate of urban tumours and 18.50% of the incidence rate of rural tumours. Lung cancer mortality accounts for 27.05% and 22.42% of urban and rural tumour mortality, respectively [18]. Conventional chemotherapy has a 25% to 35% near-term remission rate for advanced non-small-cell lung cancer (NSCLC), a median survival time of 8 to 11 months, a one-year survival rate of only 30%, and an overall 5-year survival rate of less than 2% [19].

The article "The Effect of Gefitinib on Treatment Necessity and Prognosis of NSCLC Patients with Early EGFR Mutations" was published in 2022. Journal: Contrast Media Mol Imaging.

With the understanding of the biological behaviour of lung cancer and the development of molecularly targeted therapies, the efficacy of treatment for some screened NSCLC patients has improved significantly. The most frequently detected mutations in clinical practice include EGFR and ALK mutations. For EGFR-sensitive mutations, clinical options include gefitinib, erlotinib, and erlotinib. Crizotinib has shown good efficacy against ALK mutations.

The results of this study showed that women were more likely to develop lung cancer than men *P*=0.002, and those with a long history of smoking or second-hand smoke were more likely to develop cancer *P*=0.007, which is consistent with the results of the study [20]. In the comparison of tumour recurrence rates, we found a higher recurrence rate in the experimental group (66.00%) than in the control group (40.91%), with a statistically significant difference between the two groups (*χ*^2^ = 5.937, *P*=0.015), suggesting that our patients with amplified EGFR genes were more prone to recurrence and metastasis. Interestingly, in a subgroup analysis of patients in the experimental group taking drugs versus those not taking drugs, the recurrence rate in patients with a positive EGFR gene mutation and not receiving gefitinib was 80.65%; in contrast, the recurrence rate in patients with a positive mutation and taking oral targeted drugs was 42.11%, with a difference between the two groups (*χ*^2^ = 7.797, *P*=0.005). This phenomenon corroborates with the study by Kobayashi et al. who concluded that EGFR-positive lung nodules grow faster, while EGFR-negative nodules grow relatively slowly. In the current understanding, we venture to speculate that tumour recurrence may also be genetically driven and that it is due to genetic mutations that drive the probability of recurrence in drug-ineffective patients to 80.65%. This may need to be studied by more scholars in a multicentre setting [21].

In the exploration of tumour recurrence sites we found that among the three types with high mutation frequency, i.e., exon 19 deletion, exon 20 T790M, and exon 21 L858, there was a significant difference between the different mutation types and metastasis sites (*χ*^2^ = 18.504, *P*=0.005), with a higher proportion of bone metastases occurring in exon 19 deletion (68.18%), with a higher proportion of brain metastases occurring in exon 20 T790M (56.00%), a result that suggests that we can prioritise the drug axitinib, which is more advantageous in brain metastases, to prevent brain metastases in clinical decision-making when patients with Exon 20 T790M mutations, a result that indirectly confirms the need for postoperative chemotherapy in EGFR mutation-positive patients as proposed in the study [22] and adjuvant treatment with octitinib. In subsequent survival analysis, we found that the shortest mean survival time was 43.9 months for patients in the experimental group who did not take the drug, while the mean survival time for patients in the experimental group who took the drug was 61.951 months; the control group had an intermediate mean survival time of 54.836 months, with a significant difference between the three groups (*χ*^2^ = 6.791, *P*=0.034 < 0.05). When comparing the mean survival time and 5-year survival rate for the three genes with high mutation probabilities, the highest mean survival time was found for the L858 mutation in exon 21 (62.367 months), the next highest for the deletion mutation in exon 19 (58.283 months) and the shortest for exon 20 T790M (42.936 months), and the 5-year survival rates for the three differed (*χ*^2^ = 6.095, *P*=0.047). The presence of this result further supports our hypothesis that lung cancer patients are more likely to recur and metastasise when genetically driven, and less likely to recur and metastasise and survive longer when pharmacological interventions are used. In conducting the study, we found the same view as the team in [23, 24]. So do early-stage lung cancer patients take targeted drugs as adjuvant therapy in the presence of gene drives? This is a question we may need to rethink.

The article "The Effect of Gefitinib on Treatment Necessity and Prognosis of NSCLC Patients with Early EGFR Mutations" was published in 2022. Journal: Contrast Media Mol Imaging.

In conclusion, this study suggests that early driver-positive lung cancer has a much higher probability of recurrence and metastasis and a shorter survival time in the absence of drug intervention. However, the present study is a single-centre study with undeniable limitations, and there is a greater need for a multicentre prospective study to further corroborate the findings.

## Figures and Tables

**Figure 1:** Survival curve under drug intervention.

**Figure 2:** Survival curves of different EGFR mutation types.

**Table 1:** Clinical features.

—	Name	No recurrence *n* (%)	Recurrence *n* (%)	*χ* ^2^	*P*
Gender	Male	26 (63.41)	15 (36.59)	9.148	0.002
	Female	17 (32.08)	36 (67.92)		

Age	Under 60 years old	22 (40.00)	33 (60.00)	1.763	0.184
	60 years old and above	21 (53.85)	18 (46.15)		

Alcohol consumption	No	28 (50.91)	27 (49.09)	1.425	0.233
	Yes	15 (38.46)	24 (61.54)		

Smoking	No	32 (57.14)	24 (42.86)	7.251	0.007
	Yes	11 (28.95)	27 (71.05)		

Family medical history	No	29 (48.33)	31 (51.67)	0.448	0.503
	Yes	14 (41.18)	20 (58.82)		

**Table 2:** Comparison of recurrence rate between experimental group and control group.

Groups	—	No recurrence	Recurrence	*χ* ^2^	*P*
Control group	—	26 (59.09)	18 (40.91)	5.937	0.015
Experimental group	—	17 (34.00)	33 (66.00)		
Experimental group	Not taking medication	6 (19.35)	25 (80.65)	7.797	0.005
	Taking medication	11 (57.89)	8 (42.11)		

The article "The Effect of Gefitinib on Treatment Necessity and Prognosis of NSCLC Patients with Early EGFR Mutations" was published in 2022. Journal: Contrast Media Mol Imaging.

**Table 3:** Comparison between EGFR mutation types and metastatic sites.

EGFR mutation type	Lung metastasis	Liver metastasis	Bone metastasis	Brain metastasis	*χ* ^2^	*P*
Exon 19 deletion	2 (9.09)	2 (9.09)	15 (68.18)	3 (13.64)	18.504	0.005
Exon 20 T790M	5 (20.00)	2 (8.00)	4 (16.00)	14 (56.00)		
Exon 21 L858	0 (0.00)	1 (33.33)	2 (66.67)	0 (0.00)		

**Table 4:** Means and medians of survival analysis times.

Take your medication	Average value^a^				Median			
	Estimate	Standard error	95% confidence interval		Estimate	Standard error	95% confidence interval	
			Lower limit	Upper limit			Lower limit	Upper limit
Not taking medication	43.900	3.886	36.283	51.517	46.100	5.209	35.890	56.310
Take medication	61.951	2.340	57.365	66.538	—	—	—	—
Control group	54.836	2.756	49.435	60.238	—	—	—	—
Overall	52.961	2.027	48.988	56.934	60.700	—	—	—

^a^If the survival analysis time has been checked, then the estimate will be limited to the maximum survival analysis time.

**Table 5:** Overall comparison.

—	Cardinality	Degrees of freedom	Significance
Log rank (Mantel-Cox)	6.791	2	0.034

Equivalence tests of survival analysis distributions were performed for different levels of experimental subgroups.

**Table 6:** Means and medians of survival analysis times.

Take your medication	Average value^b^				Median			
	Estimate	Standard error	95% confidence interval		Estimate	Standard error	95% confidence interval	
			Lower limit	Upper limit			Lower limit	Upper limit
Exon 19 deletion	58.283	3.342	51.733	64.833	—	—	—	—
Exon 20 T790M	42.936	4.366	34.378	51.494	44.500	6.578	31.607	57.393
Exon 21 L858	62.367	1.660	59.113	65.621	—	—	—	—
Overall	51.140	2.898	45.461	56.820	53.600	—	—	—

^a^EGFR mutation = positive. ^b^If the survival analysis time has been checked, then the estimate will be limited to the maximum survival analysis time.

**Table 7:** Overall comparison.

-	Cardinality	Degrees of freedom	Significance
Log rank (Mantel-Cox)	6.095	2	0.047

Equivalence tests for the distribution of survival analysis were performed for different levels of EFGR mutation types. ^a^EGFR mutation = positive.

## Data Availability

The figures and tables used to support the findings of this study are included in the article.
